# Small Molecule Kaempferol Promotes Insulin Sensitivity and Preserved Pancreatic ***β***-Cell Mass in Middle-Aged Obese Diabetic Mice

This article has been retracted.

**DOI:** 10.1155/2015/532984

**Published:** 2015-05-07

**Authors:** Hana Alkhalidy, William Moore, Yanling Zhang, Ryan McMillan, Aihua Wang, Mostafa Ali, Kyung-Shin Suh, Wei Zhen, Zhiyong Cheng, Zhenquan Jia, Matthew Hulver, Dongmin Liu

**Affiliations:** ^1^Department of Human Nutrition, Foods & Exercise, College of Agriculture and Life Sciences, Virginia Tech, Blacksburg, VA 24061, USA; ^2^The Metabolic Phenotyping Core, Virginia Tech, Blacksburg, VA 24061, USA; ^3^Department of Biology, The University of North Carolina at Greensboro, Greensboro, NC 27412, USA

## Abstract

Insulin resistance and a progressive decline in functional *β*-cell mass are hallmarks of developing type 2 diabetes (T2D). Thus, searching for natural, low-cost compounds to target these two defects could be a promising strategy to prevent the pathogenesis of T2D. Here, we show that dietary intake of flavonol kaempferol (0.05% in the diet) significantly ameliorated hyperglycemia, hyperinsulinemia, and circulating lipid profile, which were associated with the improved peripheral insulin sensitivity in middle-aged obese mice fed a high-fat (HF) diet. Kaempferol treatment reversed HF diet impaired glucose transport-4 (Glut4) and AMP-dependent protein kinase (AMPK) expression in both muscle and adipose tissues from obese mice.* In vitro*, kaempferol increased lipolysis and prevented high fatty acid-impaired glucose uptake, glycogen synthesis, AMPK activity, and Glut4 expression in skeletal muscle cells. Using another mouse model of T2D generated by HF diet feeding and low doses of streptozotocin injection, we found that kaempferol treatment significantly improved hyperglycemia, glucose tolerance, and blood insulin levels in obese diabetic mice, which are associated with the improved islet *β*-cell mass. These results demonstrate that kaempferol may be a naturally occurring anti-diabetic agent by improving peripheral insulin sensitivity and protecting against pancreatic *β*-cell dysfunction.

## 1. Introduction

Diabetes mellitus is a growing public health concern, presently affecting 25.8 million or 8.3% of the American population [1] and nearly 387 million people worldwide [2]. While the availability of novel drugs, techniques, and surgical intervention has improved the survival rate of individuals with diabetes, the prevalence of diabetes is still rising in the United States, with the number of people with diabetes projected to double by 2025 [3]. T2D is a result of chronic insulin resistance and loss of *β*-cell mass and function [4]. Both in experimental animals and people, obesity is a leading pathogenic factor for developing insulin resistance, which is always associated with the impairment in energy metabolism, causing increased intracellular fat content in skeletal muscle, liver, fat, and pancreatic islets. Constant insulin resistance will progress to T2D when *β*-cells are unable to secrete adequate amount of insulin to compensate for decreased insulin sensitivity, which is largely due to insulin secretory dysfunction and significant loss of functional *β*-cells [4–8]. Indeed, those individuals with T2D always manifest increased *β*-cell apoptosis and reduced *β*-cell mass [6, 7, 9]. As such, the search for novel agents that simultaneously promote insulin sensitivity and *β*-cell survival may provide a more effective strategy to prevent the onset of diabetes [10].

Recently, naturally occurring polyphenolic compounds have been the focal point of medicinal research interest due to their pharmacological implications associated with human disease with considerable attention devoted to managing diabetes [11, 12]. Polyphenols exist naturally as secondary plant metabolites and are the largest source of human dietary antioxidants, with a typical daily intake of roughly 1 g/day [13]. One of the most common polyphenolic subclasses is flavonols [14]. Kaempferol (3,5,7-trihydroxy-2-(4-hydroxyphenyl)-4H-1-benzopyran-4-one) is a flavonol, of low molecular weight (286.2 g/moL), that has been identified in many plants used in traditional medicine, including* Equisetum* spp.,* Sophora japonica*, and* Ginkgo biloba*, and edible plants, including beans, broccoli, cabbage, gooseberries, grapes, kale, strawberries, tea, and tomatoes [15, 16]. Dietary intake of kaempferol containing foods has been epidemiologically associated with a reduced risk of certain cancers and cardiovascular diseases [15]. It has been reported that kaempferol has antioxidative [17], antimicrobial [15], anti-inflammatory [18], lipolytic [19], and anticancer [20, 21] effects. However, to date, the studies regarding its effect on the pathogenesis of diabetes are very limited.

We recently demonstrated that kaempferol treatment prevented apoptosis and improved insulin biosynthesis and secretion in *β*-cells and human islets exposed to chronic hyperlipidemia [12]. Past studies have established that sustained hyperlipidemia in obese individuals plays an important role in causing *β*-cell apoptosis and dysfunction, thereby contributing to the deterioration of glycemic control and the overt development of T2D [22–24]. This study was conducted to investigate whether long-term dietary intake of kaempferol can promote metabolic homeostasis and thereby prevent diabetic pathogenesis. We show here that dietary intake of kaempferol for 5 months (mo) improved insulin sensitivity and glucose tolerances, which were associated with increased Glut4 and AMPK*α* expression in muscle and adipose tissues in middle-aged mice fed a high-fat (HF) diet.* In vitro*, kaempferol increased lipolysis and restored chronic high fatty acid-impaired glucose uptake and glycogen synthesis in skeletal muscle cells, which were associated with improved AMPK*α* activity and Glut4 expression. In addition, dietary kaempferol treatment preserved functional pancreatic *β*-cell mass and prevented hyperglycemia and glucose intolerance in STZ-induced diabetic mice. These results suggest that kaempferol may be a naturally occurring antidiabetic agent.

## 2. Methods

### 2.1. Animal Studies

Male (10-month-old) C57BL/6J mice (NCI, NIH) were individually housed in an animal room maintained on a 12-hour light/dark cycle under constant temperature (22–25°C) with* ad libitum* access to food and water. After 1 week of environment acclimation, we conducted the following two animal studies. The Institutional Animal Care and Use Committee at Virginia Tech approved the animal study protocols.

### 2.2. High-Fat Diet-Induced Obese Mice

Mice were divided into 4 groups (*n* = 12 mice/group) with blood glucose and body weight balanced and then fed a standard chow (SD) diet, with 10% of calories derived from fat, a HF diet (Research Diets Inc., New Brunswick, NJ) with 58% of calories from fat, or HF diet supplemented with kaempferol (0.01% or 0.05%) for 5 mo. Body weight and food intake were recorded weekly throughout the study. To assess fasting blood glucose, mice were fasted for 12 h, and blood glucose was measured in tail vein blood samples using a glucometer (Kroger, Cincinnati, OH). After 5 mo of dietary treatment, body composition was evaluated using an LF-90 instrument (Bruker Optics, Inc., Billerica, MA). The LF-90 body composition instrument is based on Time Domain nuclear magnetic resonance (TD-NMR) technology, which provides an* in vivo* measurement of lean tissue, body fat, and body fluid in live mice without anesthesia. Following this procedure, glucose and insulin tolerance tests were performed. For the glucose tolerance tests (GTT), mice were fasted for 12 h and injected intraperitoneally (ip) with a single bolus of glucose (2 g/kg BW). Glucose levels were measured at time points of 0, 15, 30, 60, and 120 min after glucose administration. For the insulin tolerance tests (ITT), mice were injected ip with insulin (0.75 units/kg BW), and blood glucose levels were measured at 0, 15, 30, 60, and 120 min after insulin administration. Area under the curve (AUC) was calculated using the trapezoidal rule. At the end of the study, the mice were fasted overnight and euthanized, immediately followed by the collection of blood samples. Fasting plasma total cholesterol, HDL-cholesterol, and triacylglycerol were measured by enzymatic methods using a Pointer 180 Analyzer (Pointe Scientific, Canton, MI) as described previously [25]. Plasma insulin levels were measured using a mouse insulin ELISA kit (Mercodia, Inc., Uppsala, Sweden). Blood HbA1c levels were determined using an assay kit (Henry Schein, Inc., Melville, NY). At the end of feeding experiment, mice were sacrificed and extensor digitorum longus muscle and abdominal adipose tissues were collected, snap-frozen in liquid nitrogen, and then stored at −80°C for the Western blot analyses. In a separate experiment, mice were divided into 3 groups (*n* = 8 mice/group) and fed a SD diet or SD diet containing kaempferol (0.01% or 0.05%) for 3 mo. Body weight and food intake were recorded weekly. Fasting and nonfasting blood glucose levels were measured biweekly. At the end of 3 mo, GTT and ITT were performed.

### 2.3. Streptozotocin- (STZ-) Induced Diabetic Mice

For this study, 10-month-old male mice (NCI, NIH) were divided into 3 groups (*n* = 10 mice/group) with initial fasting blood glucose and body weights balanced among groups. Mice were then fed a SD diet, a HF diet (58 kcal% fat), or HF diet containing 0.05% kaempferol. After 6 weeks of dietary kaempferol supplementation, GTT, ITT, and body composition were evaluated as described above. After this procedure, mice received ip injections of STZ dissolved in 0.1 M cold sterile sodium citrate buffer (pH 4.5) at 45 mg/kg daily for 3 consecutive days. Control mice received ip injections of saline. Body weight, food intake, and nonfasting and fasting blood glucose were measured biweekly throughout the study. Plasma insulin measurements were as stated above.

### 2.4. Immunohistochemistry

At the end of experiment, mice were euthanized, and the pancreata were dissected, weighed, and then fixed in 4% (vol/vol) formaldehyde buffer (pH 7.2). Pancreas samples were embedded in paraffin and sectioned by AML Laboratories Inc. (Baltimore, MD). A series of tissue sections (5 *μ*m thickness at 200 *μ*m interval) were prepared, mounted on glass slides, and immunofluorescently stained with an insulin antibody and FITC-conjugated secondary antibody (Abcam, Cambridge, MA) for determining *β*-cell mass. Pancreatic *β*-cell area was measured using images acquired from insulin-stained pancreatic sections. Pancreatic *β*-cell mass was calculated by dividing the area of insulin-positive cells by the total area of pancreatic tissue and multiplied by the pancreas weight [25, 26]. Four pancreatic sections from 5 mice in each treatment group were evaluated.

### 2.5. Measurements of Pancreatic Insulin Content

Pancreata were rapidly excised and weighed. Insulin was then extracted from pancreas homogenates with acid-ethanol [75% ethanol, 25% acetic acid (25% vol/vol)] overnight at 4°C. The homogenates were centrifuged (10 min, 2,000 g, 4°C) and the supernatants were neutralized with Tris buffer. Pancreatic insulin content was measured by ELISA and then normalized to the protein concentration in the same sample.

### 2.6. Cell Culture

The C2C12 mouse cells (American Type Culture Collection, Manassas, VA) were grown at 37°C and 5% CO_2_ in Dulbecco's Modified Eagle's Medium (DMEM), supplemented with penicillin (50 IU/mL), streptomycin (50 *μ*g/mL), and 10% fetal bovine serum (FBS). The cells were grown to 75% confluence and the growth medium was then switched to DMEM supplemented with 2% horse serum and penicillin (50 IU/mL) and streptomycin (50 *μ*g/mL) for differentiation.

### 2.7. Glucose Uptake Assay

C2C12 myoblasts were grown to ~80% confluence in DMEM and then differentiated for 5 days in DMEM supplemented with 2% horse serum. On day 5, the myotubes were treated for 24 h with 10 *μ*M kaempferol or vehicle (DMSO) along with a mixture of fatty acids or vehicle (BSA). The fatty acid mixture contained a 2 : 1 ratio of palmitate to oleate for a final concentration of 0.4 mM complexed with 0.4% BSA in serum-free, low glucose DMEM. Following the fatty acid and kaempferol treatment, glucose uptake was assessed in Krebs-Ringer HEPES buffer (in mM: 136 NaCl, 4.7 KCl, 1.25 MgSO_4_, 1.2 CaCl, and 20 HEPES, pH 7.4) with the addition of 10 *μ*M 2-deoxyglucose and 1.25 uCi/mL 2-deoxy-[3H]glucose. After 15 min of incubation, plates were placed on ice, washed three times with ice-cold PBS, and harvested in 400 *μ*L of 0.2 M NaOH for cell lysis. Glucose uptake was calculated based on specific activity and expressed relative to protein content.

### 2.8. Glycogen Synthesis

C2C12 myotubes were treated for 24 h with 10 *μ*M kaempferol or vehicle (DMSO) along with 0.4 mM fatty acid (FA) cocktail or BSA as stated above. After 24 h with FA and kaempferol treatment, cells were further incubated with 1.25 uCi/mL^14^C glucose (American Radiolabeled Chemicals, Saint Louis, MO) in the presence or absence of insulin (100 NM; Eli Lilly, Indianapolis, IN) for 3 h. Following this treatment, cells were rinsed twice with PBS at 4°C followed by solubilization by adding 250 *μ*L of 30% KOH. The samples were then mixed with 35 *μ*L of 60 mg/mL glycogen (Sigma-Aldrich, St. Louis, MO) in distilled water and heated at 80°C for 20 min. Glycogen in the samples was precipitated with ice-cold ethanol. Following centrifugation at 4°C (10,000 rpm) for 20 min, the pellet was collected and washed with 70% ethanol and then resuspended in 500 *μ*L distilled water. After 20 min of shaking, the glycogen precipitate was counted for the presence of ^14^C by liquid scintillation (LS 6500, Beckman Coulter, Brea, CA). Glycogen synthesis was calculated based on specific activity and was expressed relative to protein content.

### 2.9. Lipolysis Assay

C2C12 muscle cells were preincubated with kaempferol or vehicle (DMSO) for 30 min followed by addition of 20 mM glucose and 0.5 mM palmitate for 24 h. Glycerol released into the medium was then measured by using a free glycerol determination kit (Sigma-Aldrich, St. Louis, MO).

### 2.10. Western Blot Analysis

Animal tissues or cultured cells were homogenized in lysis buffer (50 mM HEPES, 0.1% (v/v) Triton X-100, 1 mM PMSF, 10 mM E-64, 10 mM pepstatin A, 10 mM TLCK, 100 mM leupeptin, pH 7.4). Supernatants of cultured muscle cell or mouse tissue lysates were collected, and protein content was measured using an assay kit. Equal amounts of protein extracts from mouse tissues or cells were subjected to Western blot analysis as described previously [27]. Nitrocellulose membranes were probed with antibody against Glut4, AMPK*α*, or phospho-AMPK*α* (Cell Signaling, Danvers, MA). The immunoreactive proteins were detected by chemiluminescence (Thermo Fischer, Rockford, IL). Nitrocellulose membranes were then stripped and reprobed with *β*-actin (animal tissues) or AMPK*α* (culture cells). The protein bands were digitally imaged for densitometric quantitation with a software program (Image J, NIH). All proteins levels were normalized to those of *β*-actin or total AMPK*α*, where applicable, from the same samples.

### 2.11. Statistical Analysis

Data were analyzed with one-way ANOVA, using Sigmaplot software program, and are expressed as mean ± standard error (SE) or mean ± standard error of mean (SEM) [28], where applicable. Treatment differences were subjected to Duncan's multiple comparison tests. Differences were considered significant at *p* < 0.05.

## 3. Results

### 3.1. Long-Term Dietary Intake of Kaempferol Reduced Body Weight Gain and Improved Body Composition and Plasma Lipid Profile in HF Diet-Induced Middle-Aged Obese Mice

In this study, we tested the metabolic effects of the long-term dietary supplementation of kaempferol (0.01% or 0.05% in the diet) in middle-aged mice fed a HF diet. The HF diet decreased the accumulative average food intake, but kaempferol supplementation for 5 mo did not alter the food consumption compared with HF diet-fed mice (Figure 1(a)). Five mo of consuming HF diet significantly increased body weight of mice. However, dietary intake of 0.05% kaempferol significantly ameliorated HF diet-induced body weight gain (Figure 1(b)). Consistently, mice fed the HF diet developed obesity as determined by measuring their relative percentage of fat (Figure 1(c)) and muscle mass (Figure 1(d)). However, kaempferol treatment had no significant effect on adiposity of obese mice. Fasting blood levels of cholesterol (Figure 1(e)), LDL-cholesterol (Figure 1(f)), and triglyceride (Figure 1(g)) were increased in HF diet-fed obese mice, which were significantly reduced by dietary intake of kaempferol. However, total cholesterol levels in kaempferol-fed mice were still significantly higher as compared to chow diet-fed mice. Fasting plasma HDL-cholesterol concentrations were increased by HF feeding but were not further altered by kaempferol treatment (Figure 1(h)). In another study to determine whether kaempferol also improves metabolism and health of SD diet-fed older adult mice, we found that dietary intake of either 0.01% kaempferol (K1) or 0.05% kaempferol (K2) for 3 mo had no effects on body weight gain (5.9 ± 0.5, 6.1 ± 0.4, and 6.0 ± 0.6 g for control, K1, and K2 group, resp.), food intake (4.25, 4.27, and 4.23 g/d/mouse), fasting (136.4 ± 4.1, 131.6 ± 3.4, and 127.9 ± 5.8 mg/dL) and nonfasting (185.4 ± 11.1, 180.5 ± 5.5, and 174.4 ± 12.2) blood glucose levels, glucose tolerance (32672 ± 1653, 31411 ± 1582, and 31078 ± 1634 AUC), and insulin sensitivity (11073 ± 1065, 10897 ± 9887, and 10574 ± 1141 AUC). Given these results, these mice were not further studied and therefore euthanized.

### 3.2. Long-Term Provision of Kaempferol Maintained Blood Glucose Homeostasis and Insulin Sensitivity in Middle-Aged Obese Mice

After 2 mo of HF diet consumption, mice displayed hyperglycemia throughout this study, as shown by persistently over 50% higher circulating glucose levels as compared with mice that consumed the SD diet. Kaempferol supplementation at this point nonsignificantly reduced the HF diet-induced rise in blood glucose. After 3 mo, however, mice fed HF diet supplemented with kaempferol exhibited significantly lower blood glucose levels than those in HF-fed mice; after 5 mo of treatment, mice fed kaempferol-supplemented diet still had significantly lower blood glucose levels (140 ± 10.5 mg/dL) as compared to HF diet-fed mice (197 ± 10.5 mg/dL), which were almost reduced to the levels shown in SD-fed mice (123.0 ± 4.8 mg/dL) (Figure 2(a)). We then performed a GTT. Data showed that kaempferol (0.05% in the diet) nonsignificantly improved glucose tolerance as demonstrated by lower blood glucose levels at 30 and 60 min (Figure 2(b)) as well as reduced AUC (Figure 2(c)) following ip glucose injection compared to HF-fed mice. Consistently, blood levels of HbA1c, which reflect an average of blood glucose over a period of two to three mo [29], were significantly lower in kaempferol-treated mice as compared to those in HF diet-fed mice (Figure 2(d)). Insulin resistance is important to the etiology of T2D and usually occurs in obesity. To determine if dietary intake of kaempferol improves insulin sensitivity in obese mice, we performed an ip ITT. As expected, HF diet treatment impaired whole body insulin sensitivity. However, dietary provision of kaempferol as low as 0.01% significantly improved plasma glucose levels (Figure 2(e)) and the AUC (Figure 2(f)) postinsulin injection in HF diet-fed mice, suggesting that kaempferol increases insulin sensitivity. We then measured plasma insulin levels after overnight fasting. We observed that fasting plasma insulin levels in HF mice were about 6-fold of those in mice that received the SD diet, suggesting that obese mice are insulin resistant (Figure 2(g)). However, plasma insulin levels in 0.05% kaempferol-treated mice were more than 50% lower as compared with HF-fed obese mice (Figure 2(g)). These data strongly suggest that long-term kaempferol supplementation maintained whole body insulin sensitivity in HF diet-induced obese mice.

### 3.3. Kaempferol Improves AMPK and Glut4 Expression in Skeletal Muscle and Adipose Tissues in Middle-Aged Obese Mice

Insulin resistance in adipose tissue and skeletal muscle, the primary site of glucose and fatty acid utilization, plays a major role in the development of HF diet-induced T2D. To further determine the molecular events that are associated with improved insulin sensitivity by kaempferol treatment, we measured the expression of AMPK and Glut4 in skeletal muscle and adipose tissues, which are two critical molecules regulating glucose uptake [30, 31]. Consistent with impaired peripheral insulin sensitivity, the expression of AMPK*α* and Glut4 proteins in both skeletal muscle (Figures 3(a)–3(c)) and adipose tissue (Figures 3(d)–3(f)) from HF diet-fed mice was significantly attenuated as compared to the control mice. However, treatment with kaempferol completely reversed these detrimental effects caused by feeding the mice with HF diet (Figures 3(a)–3(f)). These results further confirmed that long-term intake of kaempferol protects against developing insulin resistance in HF diet-induced obese mice.

### 3.4. Kaempferol Treatment Prevented High Fatty Acid-Impaired Glucose Uptake and Glycogen Synthesis in Skeletal Muscle Cells

As skeletal muscle is the major site for fuel metabolism, and obesity and insulin resistance are always accompanied with the impairment in energy metabolism, a leading pathogenic factor for T2D, we performed a series of* in vitro* assays to determine whether kaempferol has direct beneficial effects on glucose metabolism. In that regard, we cultured skeletal muscle cells with or without kaempferol in the presence of palmitate and oleic acid. We found that exposure of C2C12 myotubes to high fatty acids for 24 h impaired insulin-induced glucose uptake (Figure 4(a)) and glycogen synthesis (Figure 4(b)). However, these detrimental effects were partially reversed by treatment with 10 *μ*M kaempferol (Figures 4(a) and 4(b)).

### 3.5. Kaempferol Promoted Lipolysis and Recovered High Glucose and Fatty Acid-Impaired AMPK Activity and Glut4 Expression in Skeletal Muscle Cells

To further characterize metabolic and insulin sensitizing effects of kaempferol, we cultured skeletal muscle cells with or without kaempferol in the presence of high glucose (20 mM) and saturated fatty acid palmitate (0.5 mM), an* in vitro* environment that is frequently used to simulate diabetic condition* in vivo*. The results showed that kaempferol at physiologically relevant concentrations significantly improved lipolysis (Figure 5(a)) and reversed high fatty acid-impaired AMPK*α* activity (Figure 5(b)) and Glut4 protein expression (Figure 5(c)), a downstream target of activated AMPK*α* [31].

### 3.6. Dietary Intake of Kaempferol Ameliorated Hyperglycemia and Improved Insulin Levels in Middle-Aged Obese Diabetic Mice

While peripheral insulin resistance is common during obesity in rodents and people, its progression to T2D is largely due to insulin secretory dysfunction and significant apoptosis of functional *β*-cells [4–8], leading to an inability to compensate for insulin resistance. Past studies have established that sustained hyperlipidemia in obese individuals plays an important role in causing *β*-cell apoptosis and dysfunction, thereby contributing to the deterioration of glycemic control and the overt development of T2D [22–24]. We recently found that kaempferol treatment prevented apoptosis of cultured pancreatic *β*-cells exposed to chronic hyperlipidemic condition [12]. We therefore further assessed whether kaempferol can also protect pancreatic *β*-cell function, thereby preventing diabetes by using a T2D mouse model that was generated through a combination of HF diet feeding and three consecutive injections of low doses of STZ [32]. Regarding this, C57BL/6 mice (male, 10-month-old) were fed a SD diet, a HF diet, or HF diet containing 0.05% kaempferol. Consistent with the observations from the animal study described above, treatment with kaempferol for 6 weeks had no effect on body weight gain, food intake, fasting blood glucose levels, glucose intolerance, or insulin resistance of mice fed the HF diet (data not shown). After 6 weeks of dietary treatment, STZ (40 mg/kg BW) was administrated (ip) for 3 consecutive days to induce diabetes mediated by a destruction of islet *β*-cells in mice [33]. Our data showed that dietary ingestion of kaempferol significantly mitigated STZ-induced hyperglycemia in diabetic mice as determined by measuring fasting (Figure 6(a)) and nonfasting (Figure 6(b)) blood glucose levels. Consistently, kaempferol ameliorated the loss of body weight secondary to the development of diabetes [34] (data not shown). To determine if the improved glycemic control in mice fed the kaempferol-supplemented diet is the result of preserved islet function, we measured insulin levels in the plasma of the control and kaempferol-fed mice. As shown in Figure 6(c), plasma insulin levels in mice fed diet containing kaempferol were significantly greater as compared to those in nontreated diabetic mice, suggesting that kaempferol may ameliorate hyperglycemia primarily via preserving islet *β*-cell function.

### 3.7. Dietary Intake of Kaempferol Improved Islet *β*-Cell Mass and Insulin Content in Obese Diabetic Mice

Since STZ causes diabetes by destroying islet *β*-cells [35], we then examined whether kaempferol treatment preserved *β*-cell mass in diabetic mice by using an immunohistochemical technique. We observed that HF diet-fed mice exhibited greater pancreas weight as compared with the control mice (Figure 7(a)), which was not modulated by kaempferol supplementation (Figure 7(a)). However, STZ administration caused severe destruction of pancreatic *β*-cells as determined by evaluating the area of insulin positive cells (Figure 7(b)) and islet mass (Figure 7(c)), which consequently led to the reduction of pancreatic insulin content by nearly 80% (Figure 7(d)). However, dietary provision of kaempferol partially preserved islet *β*-cell mass (Figures 7(b) and 7(c)) and insulin content (Figure 7(d)) in diabetic mice.

## 4. Discussion

Kaempferol is a flavonol that is relatively abundant in various natural plants [36]. It has been reported that kaempferol elicits a number of health benefits, including antioxidative [17, 37], anti-inflammatory [18, 38], antihypertensive [39, 40], lipolytic [19, 41], and anticarcinogenic effects [20, 21, 42]. However, studies on whether this compound possesses antidiabetic properties are very limited. In this study, we tested the antidiabetic potential of this natural compound by using two mouse models and* in vitro* studies. It is worthy to note that, unlike many metabolic studies that used young adult mice, we used near middle-aged mice, which may be more clinically relevant, as T2D in humans often occurs during middle and late ages. We provide evidence that long-term dietary intake of kaempferol promoted metabolic homeostasis with the improved fasting blood glucose, HbA1c levels, insulin sensitivity, and glucose tolerance in HF diet-induced obese mice, which was associated with increased fuel metabolism, AMPK activity, and Glut4 expression in skeletal muscle cells. Further, dietary kaempferol also ameliorates hyperglycemia in STZ-induced diabetic mice by preserving functional *β*-cell mass. Importantly, these beneficial metabolic effects, elicited by dietary intake of kaempferol, are not due to alteration in food intake. Given that both insulin resistance in peripheral tissues and progressive *β*-cell loss and dysfunction are key components in the pathogenesis of T2D [4–8], kaempferol could be a low-cost and safe natural compound to promote energy metabolism and maintain glucose homeostasis by targeting these two defects.

It is well established that obesity is an important risk factor for T2D [43, 44]. Therefore, HF diets are commonly used as a strategy to induce obesity in animal models, leading to the development of metabolic disorders including hyperlipidemia, impaired insulin sensitivity and glucose tolerance, and elevated blood insulin and glucose [45–48]. Consistently, our data showed that consumption of the HF diet induced obesity and elevated plasma concentrations of triglycerides and cholesterol that are typical of obesity [45], which however were ameliorated in mice fed a HF diet containing kaempferol. Given that obesity is a leading pathogenic factor for developing insulin resistance and subsequent glucose intolerance [49], the improved insulin sensitivity and glucose homeostasis by kaempferol supplementation could be partially due to the secondary effects whereby long-term intake of kaempferol ameliorated obesity in mice fed a HF diet. While it is presently unclear how kaempferol affects lipid metabolism and body weight gain, previous studies demonstrated that several structurally similar flavonoids inhibit lipid absorption and lipogenesis [50–52]. Because food intake was not affected by long-term kaempferol supplementation, the decrease in fasting plasma cholesterol and triglycerides in the HF-fed mice could be caused by the regulation of the intestinal digestion and absorption of lipids and/or lipogenesis, which needs further investigation. As kaempferol treatment did not alter calorie intake in mice during the course of this study, it is also possible that the reduced body fat mass as well as body weight in kaempferol-fed mice is due to its effect on energy expenditure, given that obesity results from energy imbalance.

Several lines of evidence have shown that pharmacological activation of AMPK improves blood glucose homeostasis and lipid profile in insulin-resistant rodents [53]. AMPK is an energy sensing molecule highly conserved from yeast to all animals, which is increasingly recognized as a master regulator of whole body energy homeostasis [54]. AMPK is a heterotrimeric protein kinase composed of a catalytic subunit (AMPK*α*) and two regulatory subunits (*β* and *γ*) that sense low cellular energy levels by monitoring changes in the AMP : ATP ratio. AMP binding to the *γ* subunit induces a conformational change that allows AMPK*α* to be phosphorylated at its threonine residue (Thr 172) by the AMPK-activating protein kinase (LKB1). At the whole body level, AMPK integrates stress responses, nutrient and hormonal signals to the control of food intake, energy expenditure, and substrate utilization. At the cellular level, activated AMPK inhibits hepatic gluconeogenesis [55], promotes fatty acid oxidation [54], and regulates mitochondrial biogenesis [56]. In addition, activation of AMPK increases Glut4 expression and membrane translocation in skeletal muscle [31], thereby improving glucose uptake. Consistent with the impaired insulin sensitivity in HF-fed obese mice, we found that the protein levels of AMPK and Glut4 in skeletal muscle and adipose tissue from these animals were also considerably attenuated. However, these detrimental effects were completely reversed by supplementation of 0.05% kaempferol in the HF diet. These results suggest that kaempferol may increase peripheral insulin sensitivity via the AMPK-mediated pathway.

Both in experimental animals and people, obesity-related insulin resistance is always associated with the dysfunctions of several metabolic pathways including reduced lipolysis, fatty acid oxidation, glucose uptake, and glycogen synthesis coupled with increased glucose output [49]. Specifically, it is believed that elevated intramyocellular lipid accumulation coupled with diminished lipolysis and mitochondrial lipid oxidation play a role in the development of insulin resistance in skeletal muscle [57]. Consistently, it was found that inducing lipolysis and fatty acid oxidation in muscle cells protects against lipotoxicity-induced insulin resistance [58, 59]. In the present study, we further showed that kaempferol treatment as low as 1 *μ*M augmented lipolysis and reversed chronic hyperlipidemia-impaired glucose uptake, Glut4 expression, AMPK activity, and glycogenesis in skeletal muscle cells, which provides further evidence at cellular levels that kaempferol might be an insulin sensitizing molecule by promoting energy metabolism. However, it is presently unclear how kaempferol exerts these beneficial effects in skeletal muscle cells. Kaempferol has been shown to possess antioxidant property. While we found that pharmacological doses of kaempferol (10–50 *μ*M) showed significant free radical scavenging activity as evaluated by using an oxygen radical absorbance assay, it had no such effect at 1 *μ*M. Therefore, kaempferol promotion of skeletal muscle cell function may not be due to its potential antioxidant effect. We are presently investigating how kaempferol improves energy metabolism in skeletal muscle cells.

We further explored whether kaempferol directly protects pancreatic *β*-cell function* in vivo* by using a nongenetic mouse model of T2D, which was generated by employing a combination of feeding a HF diet and administering three mild doses (40 mg/kg) of STZ that does not cause diabetes in chow-fed mice, as demonstrated in our recent study [32]. This nongenetic diabetic mouse model manifests the metabolic characteristics of human T2D, including moderate levels of hyperglycemia, hyperlipidemia, insulin resistance, impaired insulin secretion, and reduced *β*-cell mass. The results in the present study show that kaempferol partially preserved *β*-cell mass in STZ-induced diabetic mice, which could be primarily attributable to its antidiabetic action, given that diabetes was induced before kaempferol caused changes in body weight, adiposity, or other metabolic parameters. We speculate that kaempferol treatment may protect against *β*-cell apoptosis, thereby improving islet mass, given our recent observations that kaempferol promotes viability of isolated pancreatic islets exposed to chronic hyperglycemia [60] or hyperlipidemia [12].

In summary, we provide evidence that long-term dietary supplementation of kaempferol prevents HF diet-induced metabolic disorders in middle-aged obese mice. On cellular and molecular levels, kaempferol improves glycolysis, glucose uptake, glycogen synthesis, AMPK activity, and Glut4 expression in skeletal muscle. In addition, dietary supplementation of kaempferol significantly ameliorated hyperglycemia and preserved functional islet mass in old adult obese diabetic mice. These results indicate that phytonutrient kaempferol may be used as a dietary supplement to prevent metabolic disorders that are associated with obesity and aging.

## Figures and Tables

**Figure 1:** Kaempferol supplementation had no significant effects on food consumption but reduced body weight gain and fat mass in HF diet-fed middle-aged mice. (a) Food intake was recorded twice a week and the average daily food intake was calculated. (b) Body weight of the individual mouse was measured each week. Data shown are the average body weight of last week of feeding experiment. Body composition including fat mass (c) and lean mass (d) was measured following 5 mo of standard diet or HF feeding. At the end of the experiment, fasting plasma total cholesterol (e), LDL-cholesterol (f), triglycerides (g), and HDL-cholesterol (h) were measured in duplicated samples by using mouse ELISA kits. Data are shown as means ± SE (*n* = 12). ^∗^ *p* < 0.05 versus standard diet-fed mice (C); ^#^ *p* < 0.05 versus HF-fed mice. C: standard diet; HF: high-fat diet; HF + K1: HF diet containing 0.01% kaempferol; HF + K2: HF diet supplemented with 0.05% kaempferol.

**Figure 2:** Kaempferol supplementation reduced blood glucose, HbA1c, and insulin concentrations and improved insulin sensitivity in HF diet-fed mice. (a) Fasting blood glucose levels were measured at indicated time points of dietary treatment. GTT (b) and ITT (d) were performed as described in Section 2. The area under the curve (AUC) for GTT (c) and ITT (e) was calculated. (f) Plasma insulin levels were measured using an ELISA kit. Data are shown as means ± SE (*n* = 12). ^∗^ *p* < 0.05 versus SD-fed mice (C); ^#^ *p* < 0.05 versus HF-fed mice. C: standard diet; HF: high-fat diet; HF + K1: HF diet containing 0.01% kaempferol; HF + K2: HF diet supplemented with 0.05% kaempferol.

**Figure 3:** Kaempferol supplementation completely prevented the HF diet-induced decreases in AMPK*α* and Glut4 protein expression in skeletal muscle and adipose tissues of obese mice. At the end of feeding experiment, AMPK and Glut4 protein levels in whole cell lysates of skeletal muscle ((a)–(c)) and adipose tissue ((d)–(f)) of mice were measured by immunoblotting and normalized to *β*-actin content. Values are means ± SE from 4 mice per group. ^∗^ *p* < 0.05 versus standard diet-fed mice (C); ^#^ *p* < 0.05 versus HF-fed mice. C: standard diet; HF: high-fat diet; HF + K1: HF diet containing 0.01% kaempferol; HF + K2: HF diet supplemented with 0.05% kaempferol.

**Figure 4:** Kaempferol treatment reversed high fatty acid-impaired glucose uptake and glycogen synthesis in muscle cells. C2C12 myotubes were pretreated for 30 min with kaempferol (K1: 1 *μ*M; K2: 10 *μ*M) or DMSO followed by addition of 0.4 mM fatty acid mixture (FA: 2 : 1 ratio of palmitate to oleate) or vehicle (C: BSA) as stated in Section 2. 24 h later, glucose uptake (a) and insulin-stimulated glycogen synthesis (b) were measured. Data are shown as means ± SEM (*n* = 4) of duplicate or triplicated determinations each. ^∗^ *p* < 0.05 versus vehicle alone (C)-treated cells; ^&^ *p* < 0.05 versus insulin alone-treated cells; ^#^ *p* < 0.05 versus cells treated with FA and insulin.

**Figure 5:** Kaempferol promoted lipolysis and reversed high glucose and fatty acid-impaired AMPK activity and Glut4 expression in muscle cells. C2C12 muscle cells were pretreated with vehicle (C: DMSO) or kaempferol (K1: 1 *μ*M; K2: 10 *μ*M) for 24 h and then incubated in the presence or absence of 20 mM glucose and 0.5 mM palmitate (PA) for another 24 h. (a) Glycerol released into the medium was measured after 24 h. (b) The phosphorylation of AMPK*α* (p-AMPK*α*) in whole cell lysates was measured by immunoblotting and normalized to total AMPK*α*. (c) Glut4 protein expression in the cell lysates was detected and normalized to *β*-actin content. Data are means ± SE (*n* = 3). ^∗^ *p* < 0.05 versus vehicle alone (C)-treated cells; ^#^ *p* < 0.05 versus PA alone-treated cells.

**Figure 6:** Dietary intake of kaempferol ameliorated hyperglycemia in STZ-induced obese diabetic mice. Male C57BL/6 mice (10-month-old) were fed a HF diet or HF diet containing 0.05% kaempferol (HF + K) in the diet for 6 weeks prior to administration of STZ (40 mg/kg for 3 consecutive days) and continued on the same diet for 4 weeks. Age-matched mice were fed a SD diet (C). Fasting (a) and nonfasting blood glucose levels (b) were monitored biweekly throughout the study. (c) Plasma insulin levels in fasted mice were measured by ELISA. Data are means ± SE (*n* = 10–12 mice/group). ^∗^ *p* < 0.05 versus healthy control (C); ^#^ *p* < 0.05 versus STZ alone-treated mice.

**Figure 7:** Kaempferol supplementation preserved pancreatic *β*-cell mass in STZ-induced diabetic mice. (a) Pancreas from mice given a SD diet (C), HF diet and STZ administration (HF + STZ), and HF + STZ supplemented with 0.05% kaempferol (HF + STZ + K) were isolated and weighed. (b) Fixed pancreas was then sectioned and fluorescently stained with insulin. (c) The *β*-cell mass was determined as described in Section 2. Data are shown as means ± SE (*n* = 5 mice/group). (d) Insulin content in the pancreas was measured by ELISA and normalized to protein concentration in the same sample. Data are expressed as means ± SEM (*n* = 5-6 mice/group). ^∗^ *p* < 0.05 versus healthy control (C); ^#^ *p* < 0.05 versus STZ alone-treated mice.
